# Alternate Warm and Cold Therapy (AWCT) on Uricemia, Sleep, Pain, Functional Ability, and Quality of Life (USPFQoL) in Patients with Gout: A Path Forward

**DOI:** 10.1155/2022/5471575

**Published:** 2022-03-09

**Authors:** Premalatha Paulsamy, Krishnaraju Venkatesan, ShadiaHamoud Alshahrani, Fazil Ahmad, Mohamed El-Sherbiny, Vani Manoharan, Kalaiselvi Periannan, RashaElsayed Ahmed, Kousalya Prabahar, Dawit mamiru teressa

**Affiliations:** ^1^College of Nursing, Mahalah Branch for Girls King Khalid University, Abha, Asir, Saudi Arabia; ^2^Department of Pharmacology, College of Pharmacy, King Khalid University, Abha, Asir, Saudi Arabia; ^3^College of Nursing, Mahalah Branch for Girls, King Khalid University, Abha, Asir, Saudi Arabia; ^4^Department of Anesthesia Technology, College of Applied Medical Sciences in Jubail, Imam Ab-dulrahman Bin Faisal University, P.O. Box 4030, Jubail, Saudi Arabia; ^5^Department of Basic Medical Sciences, College of Medicine, Almaarefa University, P.O. Box 71666, Riyadh 11597, Saudi Arabia; ^6^Georgia CTSA, Emory University Hospital, Atlanta, GA, USA; ^7^Lecturer in Mental Health Nursing, Oxford School of Nursing & Midwifery, Faculty of Health and Life Sciences, Oxford OX3 0FL, UK; ^8^Medical Surgical Nursing, College of Nursing Tanta University, Egypt and College of Nursing, Mahalah Branch for Girls King Khalid University, Asir, Saudi Arabia; ^9^Department of Pharmacy Practice, Faculty of Pharmacy, University of Tabuk, Tabuk 71491, Saudi Arabia; ^10^Department of Chemical Engineering, College of Biological and Chemical Engineering, Addis Ababa Science and Technology University, Addis Ababa, Ethiopia

## Abstract

**Objective:**

To understand the impact of alternate warm and cold therapy (AWCT) on uricemia, sleep, pain, functional ability, and quality of life in gout patients.

**Methods:**

A quasiexperimental, nonequivalent control group, pre and posttest design was adopted among 120 gout patients. The data were collected on demographics, comorbidities, pain level, joint swelling/joint tenderness, patient global assessment of response to treatment (PGART), health-related quality of life (HRQoL) with SF-36, sleep quality by Pittsburgh Sleep Quality Index (PSQI), and serum uric acid and assessed. Descriptive and inferential statistics were used to analyze the data.

**Results:**

Patients had mean age of 58 and 61 years, mean number of comorbidities was 1.8 and 1.4, as well as presence of arthritic comorbidities except gout was 1.1 and 0.8 among study and control group participants, respectively. Pain (*p* < 0.001), PGART (*p*=−0.01), HRQoL, sleep quality, and level of SUA (mg/dl) improved significantly (*p* < 0.01) among the study group over study periods. It affirms that the AWCT is effective in reducing pain, functional disability, and SUA, as well as improving the sleep quality and HRQoL of the gout patients. There was a reduced incidence of gout flares (*p* < 0.001), and taking additional medicines for pain (*p* < 0.01) was statistically significant among study participants. Except social functioning, other domains of health were significantly (*p* < 0.05) affected by the comorbidities like hypertension, diabetes, heart disease, renal disease, and asthma/chronic obstructive pulmonary disease.

**Conclusions:**

Gout is independently associated with higher medical and arthritic comorbidity, and AWCT can be better and cost-effective alternative therapy for gout patients. In addition, it may lead to improved cardiac function, hypertension, and renal insufficiency.

## 1. Introduction

Gout is the most common form of inflammatory arthritis globally which is a metabolic disease marked by recurrent episodes of acute arthritis caused by inflammation caused by the formation, deposition, and release of monosodium urate crystals in one or more extremity joints [1–3]. It is the most common type of inflammatory joint disease in men over the age of 40, and it can affect women after menopause [4, 5]. Epidemiologic studies confirm a global distribution [5], with an estimated prevalence of 5.1 million people in the United States [6].

Gout is a common chronic crystal deposition disorder that affects 1–6.8% of the population, depending on the population studied. Serum uric acid (SUA) levels have been found to be high throughout the world, including the Philippines and Seychelles: 25%, USA: 21–22%, Japan: 20–26%, Indonesia: 18%, Russia and Nigeria: 17%, Brazil: 13%, Turkey: 12%, Taiwan: 10–52%, Thailand: 9–11%, Mexico: 11%, Sweden: 10–16%, Italy: 9–12%, Iran and Saudi Arabia: 8%, China: 6–25%, Spain: 5–11%, and South Korea: 5–25.8% [7].

Over the last 5–10 years, hospitalizations for gout have increased by 50–100% in the United Kingdom, the United States, and Sweden [8–11]. In these countries, gout now induces more hospitalizations than rheumatoid arthritis, and hospitalizations for gout increased more than for other rheumatological conditions between 2007 and 2012 [8].

The prevalence of self-reported, health professional diagnosed gout was 3.9% in the 2015–2016 National Health and Nutrition Examination Survey (NHANES), a stratified, multistage sample representative of the U.S. adult population [12]. Gout is also commonly associated with comorbidities such as cardiovascular disease (CVD), chronic kidney disease (CKD), obesity, and other conditions. As per a retrospective study in India, hyperuricemia (H.U.) was found in 33.6% of diabetics, 35.1% of hypertensives, and 34.4% of diabetic hypertensives, with the overall incidence of H.U. in patients attending screening programs being 25.8% [7].

Furthermore, cohort studies in the United States, Taiwan, and the United Kingdom have discovered that gout is linked to an increased risk of developing atrial fibrillation, obstructive sleep apnea (O.S.A.), venous thromboembolism (V.T.E.), and pulmonary embolism [13–19].The frequency of gout attacks usually increases with time in untreated patients. Hence, understanding trends in gout prevalence is critical for adequate global healthcare resource planning, not least even though gout can be “cured” with readily available and low-cost therapies.

There is a scarcity of information available on alternative therapies for the management of gout in the Indian population and its relationship with uricemia, pain, sleep, functional ability, and HRQoL. As a result, the current study was designed to evaluate the effect of alternating warm and cold therapy (AWCT) on uricemia, sleep, pain, functional ability, and quality of life (USPFQoL) gout patients: a path forward among Indian populace.

## 2. Methods

### 2.1. Research Approach and Design

For this study, quantitative research approach with a quasiexperimental, nonequivalent control group, pre and posttest design was used; only the experimental group received the intervention, while the control group received no intervention.

### 2.2. Participants and Setting

The study participants were both men and women diagnosed with gout and who were admitted as in patients for a minimum of 10 days and who agreed to participate in the study. Patients with illnesses such as open wounds and diabetic foot ulcers, peripheral vascular diseases, absence of tophi, and patients who are receiving physiotherapy were excluded from the study. The study was conducted in two orthopaedic hospitals, and one setting was used for the intervention group, and the other was for the comparison group to avoid contamination.

### 2.3. Sample Size and Sampling Process

The minimum recommended sample size was 60, as calculated by Raosoft's online sample size calculator, with a 95% confidence level and a 5% margin of error. In the first and second hospitals, 104 and 121 chronic gout patients were admitted during the study period. Among them, 120 samples were chosen by the nonprobability convenient sampling technique and distributed for experimental (60 participants) and control group (60 participants).

### 2.4. Data Collection Tools/Instruments

The data were collected on demographics and history of comorbidities, pain level using 10 points numerical scale, joint swelling/joint tenderness with a 4-point scale (0 = none to 3 = bulging beyond joint margins), and patient global assessment of response to treatment (PGART). The PGART was rated by patients using the visual analogue scale (VAS), a 15 cm horizontal line with marked anchors: 0 = very well and 100 = very poor. With these anchors, patients were asked to respond to the following: “Given all of the ways gout affects you, rate your performance on the following scale by placing a mark on the line.” The health-related quality of life (HRQoL) was assessed, and the Medical Outcomes Study Short Form-36 (SF-36) consists of eight scaled scores, which are the weighted sums of the questions in their section. Assuming that each question carries equal weight, each scale is directly transformed into a 0–100 scale. The lower the score, the greater the disability, and the higher the score, the better the health. The SF-36 is a 36-item scale that assesses eight domains of health: physical functioning (10 components), physical role limitations (four elements), bodily pain (two elements), general health perceptions (five elements), energy/vitality (four elements), social functioning (two components), emotional role limitations (three elements), and mental health (five elements). Using the Pittsburgh Sleep Quality Index (PSQI), sleep quality was assessed. Serum uric acid (uricase method) was measured. A high serum uric acid level is currently defined as a value of at least 6.8 mg per dl (405 *μ*mol per L). These data were collected based on the core domains on that outcome measures in rheumatology (OMERACT) [20].

### 2.5. Assessment

Subjects completed and returned gout symptom diaries between follow-up visits, which the investigators reviewed at the next visit. The journals contained information such as the frequency, dates, duration, and severity of flares; the joint(s) affected; medications (both prescribed and over-the-counter); and whether the gout attack required a medical office contact or visit.

### 2.6. Intervention

Control group participants received standard care and consistent advice on diet, exercise, and weight management. The intervention group was given routine care and alternate warm and cold therapy twice a day, once in the morning and once before bedtime.Coconut oil was first applied to the lower legs and feet/the affected joints in the arm. The subjects subsequently plunged their toes and then both feet/arms, into 38° water, which was then adjusted to a comfortable temperature near 42°. The basin was covered with a plastic bag, as were the participants' legs/arms up to their knees/elbows. To allow the individual to maintain a comfortable position, a blanket and a pillow was placed beneath the knees/arms and the basin. For 4 minutes, the feet/arms were immersed. The feet/arm was then applied with cold therapy for 30 s until completing 5 cycles. Then, the feet/arms were cleansed with a foaming body shampoo and cotton gloves and dried dry with a towel.The complete procedure took 30 min and comprised a 5-minute oil rub, followed by 20 minutes of AWCT. To keep the techniques as equal as feasible, all AWCT were provided by the same person.This intervention was given for 7 days during their hospitalization, and the participants were advised to follow the same in the home after discharge in 5 days/week for one month. The baseline data and post hoc after one week and one month were assessed for both the control and study groups.  Figure 1 shows the CONSORT diagram.

### 2.7. Ethical Consideration

Official permission to conduct the study and ethical approval was obtained from the Institutional Ethical Committee with ICE/LCN/2021–10 dated 20.09.2021. Consent from the participants was collected after explaining the aim of study, their role, confidentiality of the information, and their right to depart from the study. No harm certificate was obtained from an orthopaedician for the intervention. The control group also ensured that they were following the standard care protocol of the gout treatment. Confidentiality and beneficence were assured throughout the study period.

### 2.8. Statistical Analysis

The data were processed and analyzed by SPSS software using descriptive and inferential statistics. Analysis of data was by intention-to-treat. Analysis of variance was used to examine the main effects of AWCT among the two groups on the dependent variables. The *t*-test was used to compare differences between group means. Multiple regression analysis was used to examine the effect of AWCT and comorbidity on health-related quality of life in gout patients. All statistical tests used a significance of 0.05.

## 3. Results

The characteristics of study participants are given in Table 1. Most of the demographic and clinical characteristics were similar with study and control group, which is shown in the “Goodness of fit” test. Patients had a mean age of 58 and 61 years, 43 and 38 were men among study and control groups, respectively. Mean number of comorbidity was 1.8 and 1.4, as well as presence or absence of arthritic comorbidities except gout was 1.1 and 0.8 among study and control group participants, respectively.

As given in Table 2, the average pain score in baseline, after one week, and one month improved from 8.8 to 5.7 and 8.6 to 6.9 among the study and control groups, which is statistically significant at *p* < 0.001 among the study group.There were no differences between the mean values before AWCT in the score of joint swelling/joint tenderness among the control group. In the experimental group, the PGART score was decreased after the AWCT in the first week (74 (SD, 3)) and after one month (67 (SD, 6)), *p*=−0.01). Similarly, HRQoL, sleep quality, and level of serum uric acid (mg/dl) was improved significantly (*p* < 0.05) among study group participants, but there was no significant difference in the control group.

Table 3 provides the multivariable-adjusted effect of AWCT in gout patients. A multivariable model controlled the age, employment status, marital status, gender, education level, current medications, comorbidities, and arthritis comorbidity other than gout. Among the variables studied, there was a reduced incidence of gout flares (*p* < 0.001), and taking additional medicines, both prescribed and over-the-counter medications for pain (*p*=0.01), was statistically significant among study participants. The number of joint(s) affected and hospital visits was not related significantly.

The effect of comorbidities on health-related quality of life in gout patients is given in Table 4 and Figure 2. The age, employment status, marital status, gender, education level, current medications, uric acid levels, and arthritis comorbidities other than gout were all controlled in a multivariable model. In this analysis, except social functioning, other seven domains of health status such as physical functioning, physical role limitations, bodily pain, general health perceptions, energy/vitality, emotional role limitations, and mental health were significantly (*p* < 0.05) affected by the comorbidities of the participants such as hypertension, diabetes, heart disease, renal disease, and asthma/chronic obstructive pulmonary disease.

## 4. Discussion

In the present study, 225 gout patients were screened. Among them, 120 samples were chosen by the nonprobability convenient sampling technique and distributed for experimental (60 participants) and control groups (60 participants) from two hospitals. The AWCT was given seven days during hospitalization and advised to follow the same at home for one month in the study group. The participants had 1.8 and 1.4 mean comorbidity and presence or absence of arthritic comorbidities, except gout was 1.1 and 0.8 among study and control group participants. A large study looked at the temporal relationships between the occurrence of comorbidities before and after gout diagnosis using data from the U.K. Clinical Practice Research Datalink (CPRD) [21–25]. This study confirmed the well-known association of gout with subsequent CVD and renal disease and hypertension, hyperlipidaemia, CVD, and renal disease as risk factors for gout. Cohort studies from the United Kingdom, the United States, and Canada have also validated the bidirectional relationship between gout and CKD, with CKD predisposing to gout, which increases the risk of CKD progression [26–28]. These findings show that gout can lead to these comorbidities or these comorbidities leads to gout. Hence, identifying and treating gout may be an excellent strategy to prevent the occurrence of these illnesses and can help to reduce the disease burden globally.

As given in Table 2, pain (*p* < 0.001), PGART (*p*=−0.01), HRQoL, sleep quality, and level of SUA (mg/dl) improved significantly (*p* < 0.01) among study group participants, but there was no significant difference in the control group over study periods. It confirms that the AWAT effectively reduces pain, functional disability, and SUA and improves sleep quality and HRQoL in gout patients. According to Yamamoto and Nagata's study on physiological and psychological assessment of the wrapped warm footbath as a complementary nursing treatment to induce relaxation in patients with incurable cancer, the wrapped warm footbath reduced significantly sympathetic activity in hospitalized cancer patients, which can enhance relaxation and appears to provide pain relief as well as enhanced comfort [29].

Furthermore, a pilot study found a significant antihypertensive effect after 20 minutes of the steam spa. The hypotensive effect could be attributed to improved vascular endothelial function; nitric oxide produced by vascular endothelial cells causes vascular smooth muscle cells to relax [30, 31]. Though it is not the scope of the present study, this is a more significant finding as most of the study participants had the comorbidity of hypertension. This AWCT may help them reduce their blood pressure, and the effect on gout as its impact is bidirectional.

Functional disability [32], impairment of health-related quality of life (HRQoL), and increased mortality have all been reported in gout patients [33]. As a result, gout has emerged as a significant public health concern. The KING study data confirm the impact of gout on disability and provide evidence for an independent association of gout and gout-related features with functional outcome and HRQoL. This finding supports the need for better gout treatment [34]. As a nonpharmacological, safe, and simple application, footbaths can improve postmenopausal women's quality of life and prevent problems caused by insufficient sleep quality [35].

All study group patients reported significant pain relief in our preliminary investigation into whether patients receiving AWCT would report pain relief (*p* < 0.001). An increase in parasympathetic activity and a decrease in sympathetic activity would be expected to accompany pain relief-induced relaxation. The cause of the low parasympathetic activity is unknown. Still, the reduction in sympathetic nerve activity in patients may be due to the effects of soaking in warm water, alternate cold application, and tactile stimulation from massage [29]. This pain relief improved the sleep quality, functional ability, and HRQoL of the study group gout patients. However, efferent sympathetic nerve activity is increased by negative feelings in various pain disorders. Accordingly, it is supposed that the reduction in sympathetic nerve activity found in our subjects is the primary mechanism underlying both the relaxation and pain relief effects reported. Negative feelings or depression in patients, usually seen in chronic pain disorders, on the other hand, increase efferent sympathetic nerve activity. As a result, it is assumed that the decrease in sympathetic nerve activity observed in our subjects is the prime mechanism underlying both the reported improved sleep quality and pain relief effects.

Insomnia is a common sleep disorder in adults that can have various negative health effects. The total annual cost of direct and indirect insomnia healthcare costs has been estimated at USD 100 billion. Adding to the societal expenditure, insomnia harms patients' quality of life (QoL), including impaired social and occupational functioning or productivity and impaired cognition or mood. Insomnia can also worsen and increase morbidity and complications from psychological disorders like depression and have severe consequences like an increased risk of suicide [36, 37]. Hence, improving sleep quality is a significant investment in the perspective of the patients and the nation's economy.

In 85–90% of people, hyperuricemia is the major contributor to gout due to under excretion of urate. Sweat fluid comprises sodium chloride, potassium, and nitrogen metabolites like urea, ammonia, uric acid, and creatinine [38]. Besides, reduced sympathetic nerve activity results in increased renal excretory function by affecting the renal vasculature, the tubules, and the juxtaglomerular granular cells and impaired arterial baroreflex regulation. The significant reduction in SUA in the study group may be because of this effect, and AWCT increased sweat and thirst, consequently increasing fluid intake. The cold application increases the voiding sensation, thus enhancing the uric acid elimination in urine and sweat. However, further studies are required to investigate this supposition further.

## 5. Clinical Relevance

This study results can help healthcare professionals gain greater insight into alternative therapy for gout patients suffering from pain, sleep disturbance, reduced functional ability, and HRQoL. This technique can be used at home to alleviate problems, enhance their overall quality of life, and reduce healthcare costs, and this can provide an avenue for further research studies.

## 6. Conclusion

To summarize, the AWCT holds promise as a complementary intervention for inducing sleep, pain relief, and as a result, improved functional ability, HRQoL, and uric acid elimination in gout patients. As a result, the AWCT should be a proper adjuvant alternative method for gout patients. In addition, it may lead to improved cardiac function, hypertension, and renal insufficiency.

## Figures and Tables

**Figure 1:** CONSORT diagram.

**Figure 2:** Effect of comorbidities on health-related quality of life in study and control groups.

**Table 1:** Demographic and clinical data of study and control group participants.

Variables	Study group	Control group	*P* value
Age (in years), mean (SD)	58 (16)	61 (13)	<0.001
Employment status			
Employed	31	27	<0.001
Unemployed	18	19	<0.001
Retired	11	11	<0.001
Unknown	0	3	<0.001
Married	36	44	<0.001
Male	43	38	<0.001

Education level			
Less than 8th grade	25	21	<0.001
High school	8	14	<0.001
Higher secondary	13	7	<0.001
College	14	18	<0.001
Comorbidity	1.8 (1.3)	1.4 (1.7)	<0.001
Presence or absence of arthritic comorbidities except gout	1.1 (0.7)	0.8 (0.6)	<0.001

**Table 2:** Changes in the clinical data of study and control group participants over study periods.

Dependent variables: mean (SD)	Group	Baseline	1 week	1 month	*P* value

Pain score	AWCT	8.8 (0.8)	6.3 (1.1)	5.7 (0.9)	0.001
	Control	8.6 (1.2)	7.1 (1.3)	6.9 (1.02)	0.06

Joint swelling/joint tenderness	AWD	2.1 (0.4)	1.67 (0.13)	1.1 (0.3)	0.001
	Control	2.3 (0.2)	2.0 (0.7)	2.1 (0.5)	0.551

Patient global assessment of response to treatment (PGART)	AWD	81 (7)	74 (3)	67 (6)	−0.01
	Control	79 (11)	76 (9)	80 (4)	−0.971

HRQoL	AWD	57 (16)	61 (11)	69 (7)	0.01
	Control	54 (13)	57 (17)	56 (15)	0.819

Sleep quality	AWD	16 (3.1)	14 (1.8)	11 (0.5)	0.01
	Control	15.4 (4.3)	14.7 (1.8)	15.0 (0.9)	0.907

Serum uric acid (mg/dl)	AWCT	9.9 (1.4)	8.1 (0.9)	7.2 (1.1)	0.05
	Control	9.67 (2.1)	8.7 (1.8)	8.13 (2.2)	0.653

**Table 3:** Multivariable-adjusted effect of AWCT in gout patients.

	Multivariable adjusted			
	Study	Control	*P* value	Difference (%)
Incidence	2.69 (2.3–2.7)	3.52 (3.20–3.67)	0.001	34.11
No. of joint(s) affected	1.52 (1.45–1.58)	1.66 (1.27–2.05)	0.06	9.21
Taking additional prescribed and over-the-counter medicines	1.36 (1.48–1.83)	2.07 (1.82–2.33)	0.01	9.52
Hospital visits	2.08 (1.1–2.15)	2.3 (1.34–2.8)	0.21	16.21

Results are shown as mean (99% confidence intervals). Age, employment status, marital status, gender, education level, current medications, comorbidity, and arthritis comorbidity other than gout were all controlled in a multivariable model.

**Table 4:** Multivariable-adjusted effect of comorbidity on health-related quality of life in gout patients.

	Multivariable adjusted		
	Study	Control	*P* value
Physical functioning (P.F.)	51.6	47.3	0.01
Role physical (R.P.)	47.3	44.1	0.05
Bodily pain (B.P.)	49.3	43.6	0.001
General health (G.H.)	54.3	45.7	0.01
Vitality (VT)	43.9	40.8	0.05
Social functioning (S.F.)	68.3	67.9	NS
Role emotional (RE)	53.6	42.4	0.01
Mental health (MH)	73.1	66.9	0.05
Physical component summary (P.C.S.)	36.1	32.4	0.05
Mental component summary (M.C.S.)	51.8	42.1	0.01

Age, employment status, marital status, gender, education level, current medications, uric acid levels, and arthritis comorbidity other than gout were all controlled in a multivariable model.

## Data Availability

The datasets used and/or analyzed during the current study are available from the corresponding author upon request.
